The article "Fitz-Hugh-Curtis Syndrome in a Male Patient: A Case Report and Literature Review" was retracted in 2015. Reasons: duplicate publication; overlap with earlier publications.

# Fitz-Hugh-Curtis Syndrome in a Male Patient: A Case Report and Literature Review

**DOI:** 10.1155/2012/457272

**Published:** 2012-03-26

**Authors:** Shireesh Saurabh, Eric Unger, Constantinos Pavlides

**Affiliations:** ^1^Drexel University College of Medicine, Philadelphia, PA 19102, USA; ^2^Hahnemann University Hospital, Philadelphia, PA 19102, USA

## Abstract

Fitz-Hugh-Curtis syndrome is a condition characterized by inflammation of the liver capsule with concomitant pelvic inflammation without involvement of liver parenchyma. It is classically seen in young women who present with sharp, pleuritic right upper quadrant pain, usually but not always accompanied by symptoms of pelvic inflammatory disease (PID), and is frequently confused with biliary tract disease. Rarely the syndrome has been reported in males, and hematogenous and lymphatic spread to liver is thought to be the underlying mechanism. Serological tests and computed tomography (CT) scan may aid in diagnosis of Fitz-Hugh-Curtis syndrome. Definitive diagnosis is made by laparoscopy, which provides both diagnostic and therapeutic benefits. We report a case of Fitz-Hugh-Curtis syndrome in a young male patient, which was diagnosed and treated by laparoscopy. We also include a review of the literature.

## 1. Introduction

Fitz-Hugh-Curtis syndrome is an extrapelvic manifestation of pelvic inflammatory disease and is characterized by perihepatic adhesions between liver capsule and diaphragm or anterior peritoneal surface [1–3]. Most Fitz-Hugh-Curtis syndrome patients are women of child bearing age and rarely has the syndrome been reported in males. The predominant symptom is pain in the right upper quadrant, which may be confused with biliary disease. Pelvic manifestation of pelvic inflammatory disease (PID) may not be present in male patients. An abdominal computed tomography (CT) scan may reveal subcapsular enhancement of the liver in arterial phase [4]. We herein report a case of Fitz-Hugh-Curtis syndrome in a male patient that was diagnosed via laparoscopy.

## 2. Case Report

A 29-year-old African American male with Russell-Silver Dwarfism presented with one-day history of diarrhea, nausea, vomiting, right side abdominal pain, and abdominal distention. The pain was constant, gradually increasing in severity, and not related to food intake. The patient denied fever and other gastrointestinal or genitourinary complains. His medical history was significant for Russell-Silver Dwarfism, calcium deficiency, cardiomegaly, and bilateral testicular implants for undescended testicles. The patient was sexually active only with his girlfriend and denied any history of sexually transmitted disease. On examination patient was afebrile and his vitals were stable. His abdomen was soft, mildly distended and diffusely tender on right side. There was no abdominal guarding, rigidity, or rebound tenderness. Laboratory workup revealed white blood cell (WBC) count of 14,000/*μ*L with normal liver function tests. Chest and abdominal radiographs appeared normal. CT scan of the abdomen and pelvis showed a small amount of free fluid in pelvis; the proximal appendix appeared normal, however, the distal appendix was not visualized. The liver capsule appeared normal and there was no subcapsular fluid collection as seen in Figure 1.

The patient was admitted to the surgical service. He was made nil per os (NPO) and placed on intravenous fluids and pain medication. His symptoms of anorexia, diarrhea, and nausea remained unchanged. His right-sided abdominal pain worsened, while the WBC count normalized. He was refusing any surgical intervention at this point. On hospital day 5, a repeat abdominal CT scan demonstrated a normal appearing liver, small bowel, large bowel, and appendix, with a mild increase in pelvic free fluid. The clinical diagnosis at this point was abdominal pain of unknown etiology.

As the patient's symptoms did not improve with conservative management, he ultimately agreed to undergo a diagnostic laparoscopy and was taken to the operating room on hospital day 9. The cecum and the appendix appeared normal. The small bowel was run in a retrograde fashion starting at the cecum, and no stricture, mass, or perforation was noticed. The large bowel also appeared normal. There were extensive adhesions between the liver and anterior abdominal wall, as seen in Figure 2. These adhesions were lysed using the electrocautery and Endo Shears. Cultures were also obtained from the pelvic free fluid. Appendectomy was not performed as per patient's wishes. Following the procedure, the patient reported complete resolution of his symptoms. His diet was gradually advanced, which he tolerated well, and was discharged on postoperative day 2. Pelvic free fluid cultures were negative.

## 3. Discussion

Fitz-Hugh-Curtis syndrome was first described in 1920 by Carlos Stajano. In the 1930s Thomas Fitz-Hugh and Arthur Curtis also described the syndrome and made a connection between right upper quadrant pain following a pelvic infection and violin-string like perihepatic adhesions [5]. The first case of gonococcal perihepatitis in a male was reported by Kimball and Knee in 1970 [6].

The incidence ranges from 4% to 14% in women with PID, but is as high as 27% in adolescents with PID, whose less mature genitourinary tract anatomy makes them more susceptible to infection [1]. There are very few reported cases in male patients. *Neisseria gonorrhoeae* and *Chlamydia trachomatis* are thought to be the primary causative agents. There is no reported relation with Russell-Silver Dwarfism.

The pathogenesis of Fitz-Hugh-Curtis syndromes is poorly understood. In women, the inflammation of the liver capsule has been attributed to the direct bacterial spread from an infected fallopian tube via the right paracolic gutter. In men, hematogenous and lymphatic spread to liver has been postulated as the underlying mechanism of spread [1, 3].

The predominant symptoms are right upper quadrant pain, tenderness, and pleuritic right-sided chest pain [2]. These symptoms can pose diagnostic challenges as they may be confused with biliary tract symptoms. In a clinical setting, the diagnosis is adequately established by excluding other possible causes of right upper quadrant pain. On laboratory examination, white blood cell count can be elevated in nearly half of the patients, while liver function tests are normal in most patients. Because urethral cultures frequently fail to demonstrate the presence of gonorrhea and Chlamydia, the serologic microimmunofluorescence antibody test is helpful in diagnosis [2]. CT scan may show subcapsular fluid collection, thickening of hepatic capsule in the arterial phase, and wedging enhancement of the involved liver parenchyma in more than 50% of patients. In our patient, CT scan showed a normal hepatic capsule [4]. CT scan is more sensitive than ultrasound in diagnosis of Fitz-Hugh-Curtis syndrome [7]. Definitive diagnosis requires invasive procedures like laparoscopy or laparotomy.

Most cases of Fitz-Hugh-Curtis syndrome are managed with antibiotics against Gonorrhea and Chlamydia. In our case if the diagnosis had been made preoperatively, a trial of antibiotics may have been beneficial. If symptoms persist, then surgical lysis of adhesions should be considered. Laparoscopy has both diagnostic and therapeutic benefits. It provides a less invasive therapy than laparotomy. Mechanical lysis of adhesions can provide complete resolution of symptoms [8, 9].

## 4. Conclusion

Fitz-Hugh-Curtis syndrome is inflammation of liver capsule associated with genital tract infection. It occurs mostly in premenopausal women; however, cases in males have also been reported. Diagnosis is made by clinically eliminating other causes of right upper quadrant pain. Laparoscopy has both diagnostic and therapeutic benefits. Mechanical lysis of adhesions can provide complete resolution of symptoms.

## Figures and Tables

**Figure 1:** Normal appearing liver capsule and no perihepatic fluid collection.

**Figure 2:** Demonstrates extensive adhesions between liver and anterior abdominal wall (violin-string appearance).
